RETRACTED

# CNN-Based Cross-Modal Residual Network for Image Synthesis

**DOI:** 10.1155/2022/6399730

**Published:** 2022-08-10

**Authors:** Rajeev Kumar, Vaibhav Bhatnagar, Amit Jain, Mahesh Singh, Z. H. Kareem, R. Sugumar

**Affiliations:** ^1^Department of MCA, Dewan Institute of Management Studies Meerut UP, India; ^2^Department of Computer Applications, Manipal University Jaipur, India; ^3^Department of Computer Science and Engineering, Guru Nanak Dev Engineering College, Ludhiana, Punjab, India; ^4^Kebri Dehar University, Ethiopia; ^5^Medical Instrumentation Techniques Engineering Department, Al-Mustaqbal University College, Babylon, Iraq; ^6^Department of Computer Science & Engineering, Saveetha School of Engineering, Saveetha Institute of Medical and Technical Sciences, Chennai 602105, India

## Abstract

This study attempts to address the issue that present cross-modal image synthesis algorithms do not capture the spatial and structural information of human tissues effectively. As a consequence, the resulting photos include flaws including fuzzy edges and a poor signal-to-noise ratio. The authors offer a cross-sectional technique that combines residual modules with generative adversarial networks. The approach incorporates an enhanced residual initial module and attention mechanism into the generator network, reducing the number of parameters and improving the generator's feature learning capabilities. To boost discriminant performance, the discriminator employs a multiscale discriminator. A multilevel structural similarity loss is included in the loss function to improve picture contrast preservation. On the ADNI data set, the algorithm is compared to the mainstream algorithms. The experimental findings reveal that the synthetic PET image's MAE index has dropped while the SSIM and PSNR indexes have improved. The experimental findings suggest that the proposed model may maintain picture structural information while improving image quality in both visual and objective measures. The residue initial module and attention mechanism are employed to increase the generator's capacity for learning, while the multiscale discriminator is utilized to improve the model's discriminative performance. The enhanced method in this study can maintain the structure and contrast information of the picture, according to comparative experimental findings using the ADNI dataset. The produced picture is hence more aesthetically similar to the genuine print.

## 1. Introduction

With the development of science and technology, there are various ways of acquiring medical images, and different modalities of medical images have distinct advantages and disadvantages. For example, magnetic resonance imaging (MRI) has no radiation on the human body, the soft tissue structure is displayed, and rich diagnostic information can be obtained, but the acquisition time is extended, which is prone to artifacts; positron emission computed tomography (positron emission tomography (PET)) can make an early diagnosis of the disease through the functional changes of the tissue in the diseased area, but it is expensive, and the image resolution is low. Furthermore, studies have shown that the morphological or functional abnormalities of the human body caused by diseases are often manifested in various aspects. Therefore, the information obtained by a single modality imaging device usually cannot fully reflect the complex characteristics of the disease [1]. Still, clinical medical images of different modalities are collected simultaneously. It requires a lot of time and financial resources. Therefore, how to use the medical images of the existing modalities to accurately synthesize the pictures of the needed modalities through computer technology has been the research direction in recent years.

RETRACTED

The majority of medical picture cross-modality synthesis techniques are based on deep learning, which may be classified as cross-modality synthesis methods based on paired data or cross-modality synthesis methods based on unpaired data depending on the kind of data employed. This work investigates cross-modal synthesis approaches based on paired data since cross-modal synthesis based on unpaired data cannot provide subject-specific visuals. PET scans (positron emission tomography scans) are frequently performed in combination with CT scans or MRI scans (magnetic resonance imaging scans). While CT and MRI scans provide images of the inside organs and tissues of your body, PET scans can provide your doctor with a glimpse of complicated systemic disorders because they highlight cellular concerns. PET scans employ positrons as opposed to MRIs. Your body is given an injection of a tracer that enables the radiologist to view the region being scanned. While PET scans are used to examine your body's function, an MRI scan may be utilized to determine the form of your organs or blood arteries. 3D CNN was utilized in the literature [2] to predict from MRI to PET. Each sample picture was broken into many image blocks in the experiment to maximize the quantity of sample data. The method created a PET picture with an excellent classification effect. A deep residual inception encoder-decoder neural network (RIED-Net) was suggested in the literature [3] to learn the mapping between pictures of various modalities and improve generation performance. CNN-based approaches outperform older methods because they can automatically and effectively learn and pick characteristics. The transfer learning of VGG16 with one retrained ConvLayer produces the best results, which are somewhat higher than the state-of-the-art result. The specified feature may learn from the new dataset using the unfrozen ConvLayer. As a result, the specific feature is an important aspect in improving accuracy; a model's strength of expression and overfitting must be balanced. A network that is too basic frequently cannot learn enough from the data and so cannot achieve high accuracy. An extremely complicated network, on the other hand, is difficult to train and soon overfits. As a result, precision remains poor. Only a network structure with the correct size and other efficient overfit prevention strategies, such as a proper dropout rate and data augmentation, will produce the best outcomes. However, due to time constraints, further research is required. Training a fine-tuned deep convolutional neural network with defrosted ConvLayers tends to overfit in transfer learning. Other more powerful CNN models, such as ResNetv2 and ensembles of multiple CNN models, have not been evaluated, but they may improve the results; visualization should be added to improve understanding and explanation of the CNN-based system's results, as these are required for the adaptation of a CNN-based system in real clinical applications. Literature [4] suggested a context-aware generative adversarial network that uses an artificial context model to get the high-accuracy and resilient mapping from MRI to CT (computed tomography) images. A multichannel generative adversarial network was presented in the literature [5] to manufacture PET pictures. The experiment was carried out on 50 lung cancer patients' PET-CT data to produce more realistic PET pictures. To produce projected PET data with given CT data, literature [6] paired a fully convolutional network with a conditional generative adversarial network and obtained excellent results. In contrat to statistical parameter mapping analysis, literature [7] developed a 3D generative network model based on residual network to learn the mapping from MRI to FDG (fluorodeoxygloucose). Despite the excellent results of the above cross-modal synthesis approaches, owing to the complicated spatial structure of medical pictures, the above synthesis results still cannot accurately capture the edge information of human tissue, and there are issues such as poor signal-to-noise ratio and fuzzy edges. We present the Cross-Modal Contrastive Generative Adversarial Network (XMC-GAN) in “Cross-Modal Contrastive Learning for Text-to-Image Generation,” which addresses text-to-image generation by learning to maximize the similarity matrix between text and image using intermodal (image-text) and intramodal (image-image) contrastive losses. This method assists the discriminator in learning more robust and discriminative features, making XMC-GAN less prone to mode collapse even with one-stage training. In comparison to earlier multistage or hierarchical techniques, XMC-GAN provides state-of-the-art performance with a simple one-stage generation. It is trainable from start to finish and simply requires image-text pairings (as opposed to labeled segmentation or bounding box data). Furthermore, the available public medical picture data collection has very little matched data. The majority of the data utilized in the aforementioned approaches are gathered by hand, which necessitates large personnel and material resources.

RETRACTED

To summarize, this study presents a technique for the cross-modal synthesis of PET pictures from MRI images by combining residual modules and generative adversarial networks to enhance the synthesis of subject-specific PET images with little paired data. The three primary points of the main work are as follows: the generator now includes an enhanced residual initial module and an attention mechanism to completely extract the features of MRI pictures; the pix2pix network architecture has been upgraded, and the discriminator now uses a multiscale discriminator to increase discriminate performance and reduce loss; the function incorporates a multilevel structural similarity loss based on the classic adversarial loss and L1 loss, which improves picture contrast preservation.

### 1.1. Advantages and Limitations of Medical Imaging

The ability to promptly and precisely diagnose sickness and determine its severity or harmless nature is one of the potential advantages of imaging tests. It might not be essential to perform invasive diagnostic techniques such as exploratory surgery, angiography, or cardiac catheterization. Medical imaging is crucial when a person has a chronic illness or a kind of cancer, not only for the initial diagnosis but also for tracking how the illness is responding to therapy, determining whether the illness is advancing, and determining when treatment should be discontinued or changed.

One of the drawbacks of medical imaging is that there is a slight increase in the likelihood that a person exposed to X-rays would acquire cancer later in life. Cataracts, skin reddening, and hair loss are all tissue consequences that occur at quite high levels of radiation exposure and are uncommon for many types of imaging tests.

## 2. Related Work

### 2.1. Generative Adversarial Networks

The fundamental generative adversarial networks (GAN) model consists of the input vector, generator, and discriminator. The generators and discriminators are both implicit function expressions that are often employed by deep neural networks. GAN can train the predictive model of any distribution of data using adversarial approaches and get great results. GAN's primary job is to train an adversarial generator and discriminator. The objective goal is either a stronger generator or a more sensitive discriminator, depending on the project's needs. Thus, generative adversarial networks are used in CNN-based cross-modal residual networks for image synthesis. Cross-modality image estimation includes creating pictures for one form of medical imaging from those for another. It has been demonstrated that convolutional neural networks (CNNs) are effective in recognizing, classifying, and extracting picture patterns. CNNs are used as generators in generative adversarial networks (GANs), and estimated pictures are classified as true or false based on a second network. In the context of the image estimating paradigm, CNNs and GANs may be seen more broadly as deep learning techniques since imaging data frequently have a large number of network weights. The CNN/GAN image estimate literature almost exclusively uses MRI data, with PET or CT being the two main modalities. Literature [8] created the first generative adversarial network (GAN) in 2014, which included a generator *G* and a discriminator *D*. The generator takes noise *z* from distribution as input, maps it to the data space, records the data distribution of the actual sample *x*, and creates a sample *G*(*z*) that looks like the original data. The produced samples and the real samples are sent to the discriminator, and the purpose is to categorize the generated samples *G*(*z*) as false and the actual samples as true. GAN is a process in which the generator and discriminator are always in conflict, playing a game of maximum and minimum values until they strike a dynamic equilibrium. GAN's goal function is as follows:

(1) $$\begin{array}{c} \underset{G}{\min}\underset{D}{\max}V\left(D,G\right)=E_{x\sim P_{\text{data}}\left(x\right)}\left[lnD\left(x\right)\right]+E_{z\sim P_{z}\left(z\right)}\left[\ln\left(1-D\left(G\left(z\right)\right)\right)\right]. \end{array}$$

Since the results generated by the unconditional generative adversarial network have great uncertainty, literature [9] proposed to add additional information *y* to the generator and discriminator as a condition to construct a conditional generative adversarial network (CGAN). The loss function of CGAN is defined as

(2) $$\begin{array}{c} L_{\text{CGAN}}\left(G,D\right)=E_{x,y}\left[lnD\left(x,y\right)\right]+E_{x,z}\left[\ln\left(1-D\left(x,G\left(x,y\right)\right)\right)\right]. \end{array}$$

The pix2pix network [10] is a type of CGAN for image translation. However, it no longer inputs noise but directly inputs the original image as a condition to the generator. The discriminator uses the target image and the true and false image pair composed of the generated image and the original image as input to judge the true and false.

RETRACTED

### 2.2. Residual Initial Block

The structure of the initial residual block [3] is shown in Figure 1, including two paths. Among them, two 3 × 3 convolution paths extract data features. A 1 × 1 initial residual short-circuit connection can deepen (in the encoder) or reduce (in the decoder) the depth of the convolution kernel while solving the input. The problem is that feature maps and output feature maps have different channels, ensuring the fusion of input and output maps at the pixel level. Compared with the inception module, the initial residual block has fewer parameters and a more straightforward structure, which can solve the problems caused by the depth of the network.

### 2.3. Attention Module

[11] proposed an attention module for medical images; the structure is shown in Figure 2. The attention mechanism determines the attention coefficients of different regions on each input *x*^l^ by gating the signal *g*, allowing the network to focus on areas more relevant to the task and suppress irrelevant background regions. The neural network with the added attention module has higher sensitivity and accuracy

## 3. Proposed Algorithm

We have provided a generally and locally aware GAN framework for cross-modality transfer from MRI to PET in this research. To improve the quality of generated PET scans, the suggested multipath GAN architecture assists in simultaneously collecting both global structure and local texture. To assist the generative model in accurately learning the fundamental bimodal data distribution, the overall framework and the combined synthesis goal function were created. Experimental findings show that our methodology not only produces PET scans with higher-quality images. The model framework of the improved fusion residual module and generative adversarial network cross-modality PET image synthesis method is shown in Figure 3. The generator takes authentic MRI images as input, learns the feature mapping relationship between MRI and PET, and generates synthetic PET corresponding to accurate MRI synthesis.

PET and natural PET are spliced with accurate MRI to form a true and false image pair. Next, the two discriminators use the true and false image pairs as input to perform true and false discrimination. Finally, the weighted average of the two discrimination results is used as the final result.

RETRACTED

### 3.1. Generator Network

Due to its good performance and efficient use of memory, U-Net [12] is widely used in medical image segmentation tasks. Therefore, the algorithm in this paper uses U-Net as the generator.

The generator structure is shown in Figure 4, which consists of an encoding path and a decoding path. The encoding course consists of a series of 3 × 3 convolutions, 4 × 4 convolutions, batch normalization, and activation layers. The algorithm replaces the top pooling layer in U-Net with a convolution layer, continuously extracts critical features of MRI images through convolution operations, and compresses the vital information extracted from soft layers to high layers. The decoding path consists of a series of 3 × 3 convolutions, 4 × 4 deconvolutions, batch normalization layers, and activation layers and reconstructs the final output from the feature maps compressed by the encoding path.

To better learn the pixel information in the image, the algorithm in this paper introduces the improved residual initial module into the encoding and decoding paths to ensure a better generation effect. Increasing the size of the convolution kernel in the neural network can expand the receptive field, but blindly increasing the convolution kernel will increase the network parameters and bring specific difficulties to the training of the network. Therefore, the algorithm in this paper adds a 3 × 3 convolution to the 3 × 3 convolution path of the initial residual module, replaces the larger convolution kernel with 3 small convolution kernels, and reduces the receptive field as much as possible while expanding the receptive field—network parameters. In addition, the introduction of the initial residual module can also solve the problem of gradient disappearance caused by the depth of the network.

Since the structural information and spatial information of medical images are more complex than natural images, to better extract the critical structural features in MRI images, the algorithm in this paper sets the encoder-decoder path depth of the generator to 7 layers. However, considering the network complexity and memory consumption, the algorithm does not put the improved residual initial module in all convolutional layers of the encoding and decoding paths but compares the generation effect through multiple experiments and finally puts the initial residual module in the middle four layers of the network; only two 3 × 3 convolutions are used in the first 3 layers of the encoding path and the last 3 layers of the decoding path, which reduces network parameters and training time while improving the generation quality.

RETRACTED

The skip connection in U-Net can capture the contextual features from the encoding path to the decoding path. The fusion of low-level features and high-level features can retain more detailed information of high-level feature maps, but it may also contain feature information irrelevant to the synthesis task. Therefore, to improve the synthesis quality, the algorithm in this paper introduces a self-attention mechanism in the skip connection path and combines the features extracted by the decoding path before the skip connection operation. The event features through the attention gate mechanism and further eliminates the skip connection.

The interference caused by irrelevant features and noise in the MRI images highlights the critical elements in the skip connections to capture the essential information of MRI images better.

In addition, to prevent the network from overfitting, the algorithm also introduces a dropout operation in the generator. Finally, the synthesized PET image is obtained through the Tanh activation function after encoding and decoding the feature information.

### 3.2. Discriminator Network

To better learn the local and global features of PET images, improve the game ability of the discriminator, and enable the generator to generate PET images that are more in line with the actual distribution, this paper adopts multiscale discriminators, namely, local discriminator and global discriminator. With two discriminators with different receptive fields (70 × 70 and 128 × 128), the generator and discriminator can learn the relationship between the spatially shorter and longer distance pixels.

Based on the idea of patchGAN, the discriminator network first divides the image into N × N blocks and then discriminates whether each subblock is true or false. The two discriminator networks are 5 layers and 7 layers, respectively, composed of convolution layers, batch normalization layers, and activation layers alternately. Finally, the weighted average of all results is used as the output of the discriminator.

### 3.3. Loss Function

This paper uses adversarial loss, L1 loss, and multiscale structural similarity loss (MS-SSIM) as loss functions.

#### 3.3.1. Adversarial Loss

Adversarial loss can constrain the generated results to a certain extent, making the results closer to the actual distribution. The damaging loss is shown in

(3) $$\begin{array}{c} L_{\text{GAN}}=\frac{1}{N}\overset{N}{\underset{n=1}{\sum }}\left[-D\left(G\left(x,z\right)\right)\right]. \end{array}$$

#### 3.3.2. L1 Loss

The L1 loss is passed through the generator to reduce the difference between natural and synthetic images. The L1 loss is shown in

(4) $$\begin{array}{c} L_{L1}=\frac{1}{N}\overset{N}{\underset{i=1}{\sum }}\left|x_{i}-y_{i}\right|. \end{array}$$

RETRACTED

#### 3.3.3. MS-SSIM Loss

Structural similarity (SSIM) was initially described by literature [13] and proposed to measure the similarity of two images. The introduction of multiscale structural similarity loss into the loss function can better preserve the brightness and contrast information of the image.

The MS-SSIM loss is shown in equation

(5) $$\begin{array}{c} L_{\text{MS}-\text{SSIM}}\left(x,y\right)={\left[L_{M}\left(x,y\right)\right]}^{a_{M}}\overset{M}{\underset{j=1}{\prod }}{\left[c_{j}\left(x,y\right)\right]}^{\beta_{j}}{\left[s_{j}\left(x,y\right)\right]}^{\gamma_{j}}. \end{array}$$

Among them, *L*_*M*_(*x*, *y*), *c*_*j*_(*x*, *y*), and *s*_*j*_(*x*, *y*) represent the brightness, contrast, and structural similarity of the image, respectively, and *α*_*M*_, *β*_*j*_, and *γ*_*j*_ represent the weights occupied by different parts, respectively.

The final loss function of the model is as follows:

(6) $$\begin{array}{c} L=\lambda_{1}L_{\text{GAN}}+\lambda_{2}L_{L_{1}}+\lambda_{3}L_{\text{MS}-\text{SSIM}}. \end{array}$$

Among them, *λ*_*i*_(*i* = 1,2,3) is the weight coefficient of each loss.

## 4. Experimental Results and Analysis

### 4.1. Experimental Platform

The experiments in this article are run using the PyTorch framework, with an Intel i7-6700 CPU and an NVIDIA GeForce GTX1080Ti GPU as the hardware setup. The software environment consists of Ubuntu 16.04, CUDA 9.0, cuDNN 7.6, PyTorch 1.1.0, and Python 3.7.

### 4.2. Data Preparation and Parameter Setting

The Alzheimer's disease neuroimaging initiative (ADNI) public dataset [14] was utilized, with 33 problems eliminated, to create paired MRI and PET scans of 716 Alzheimer's disease participants. Subjects' aberrant data were subsequently accepted, and 683 subjects' data were eventually utilized.

Before training, data is preprocessed. The FSL software [15] is utilized for data preparation in this research, with neck removal, skull stripping, and linear registration to MNI152 space among the processes. Three-dimensional data with a size of 9110991 is acquired after preprocessing. As model input, the 40th axial slice of the 3D data was collected and upsampled to a size of 128128. The experiment uses the 5-fold cross-validation approach to get more accurate experimental findings. All of the data is split into five groups at random, with four of them serving as the training set (547 slices) and the other serving as the test set (136 pieces).

The weight coefficients of the loss function are changed throughout the network training phase. Because the input image's pixel range is (0, 1), the resultant L1 loss is much less. When the MS-SSIM loss coefficient is more important, the brightness of the synthesized picture is higher, and when the volume is lower, it has a less significant influence on the outcome. As a result, the weight of each loss function is eventually adjusted to 1 = 1, 2 = 100, and 3 = 1 after numerous testing and troubleshooting. Furthermore, the batch size is set to 16, the initial learning rate is set at 0.0002, the network is optimized using the Adam optimizer, and 200 epochs are iteratively trained. The learning rate for the first 100 epochs remains intact, whereas the learning rate for the final 100 epochs is lowered linearly to zero.

RETRACTED

### 4.3. Experimental Results

To verify the performance of the improved algorithm in this paper, this paper conducts experiments on the ADNI dataset. The algorithm uses the pix2pix model as the benchmark model and, at the same time, compares with RIED-Net, pGAN [16], and GAN with residual network [17] as the generator (ResnetGAN); the GAN model with residual U-Net as the generator [7] and other mainstream algorithms based on CNN and GAN are compared and evaluated from qualitative and quantitative aspects. A total of 5 sets of cross-experiments are carried out.

#### 4.3.1. Qualitative Evaluation

The qualitative comparison between the generated results of the algorithm in this paper and the generated results of other algorithms is shown in Figure 5. As shown from the first row of Figure 5, compared with the actual image, different algorithms have the problem of significant deviation of results and speckle noise. The consequences of this algorithm are more complete. In addition, the structural edges of the results obtained by other algorithms look too smooth or blurred. In contrast, the results generated by the algorithm in this paper are relatively more precise. The difference is also improved to a certain extent, and the visual is closer to the actual image.

In addition, due to the different brain sizes of other subjects, there is still a specific deviation after linear registration to the standard space. As shown in the second and third rows of Figure 5, pix2pix and Resnet GAN cannot learn this mapping relationship well, and the generated images and size mapping confusion. Although other algorithms can learn the change of structure size, there is a lot of missing edge information, and there are still problems of noise and significant structural errors. In contrast, the results synthesized by the algorithm in this paper have better edge integrity and no noise speckles, which may be because the improved residual initial module is introduced in this paper, which improves the model performance. It can be seen that the results generated by the improved algorithm in this paper are more diverse and can preserve the edge structure of the image more thoroughly.

RETRACTED

#### 4.3.2. Quantitative Evaluation

In this paper, mean absolute error (MAE), peak signal-to-noise ratio (PSNR), and structural similarity index (SSIM) are used as evaluation indicators.  Figure 6 shows the quantitative evaluation of MAE.

MAE [10] and PSNR [12] are calculated as

(7) $$\begin{array}{c} \text{MAE}=\frac{1}{n}\overset{n}{\underset{i=1}{\sum }}\left|y_{i}-x_{i}\right|, \end{array}$$

(8) $$\begin{array}{c} \text{LGPSNR}=10*\mathrm{lg}\left(\frac{{I_{\max}}^{2}}{\text{MSE}}\right). \end{array}$$

Among them, MSE is the mean square error of the two images, and *I*_max_ represents the maximum value of the image color, which is expressed as 255 using 8-bit sampling points.

SSIM [15] is calculated as

(9) $$\begin{array}{c} \text{SSIM}\left(x,y\right)=\frac{\left(2\mu_{x}\mu_{y}+c_{1}\right)\left(2\sigma_{xy}+c_{2}\right)}{\left(\mu_{x}^{2}+\mu_{y}^{2}+c_{1}\right)\left(\sigma_{x}^{2}+\sigma_{y}^{2}+c_{2}\right)}. \end{array}$$

Among them, *μ*_*x*_, *μ*_y_, *σ*_*x*_^2^, *σ*_*y*_^2^, and *σ*_*xy*_ are the mean, variance, and covariance of the pictures *x* and *y*, respectively; *c*_1_ = (*k*_1_*L*)^2^ and *c*_2_ = (*k*_2_*L*)^2^ are two constants that prevent the denominator from being 0.  Figure 7 shows the quantitative evaluation of PSNR.

Table 1 shows the quantitative indicators derived from the comparison experiments. The MAE indices of the results synthesized by the method in this research are all lowered when compared to previous algorithms, showing that the enhanced technique in this work is more stable. The SSIM values of the findings in this work are 0.106, 0.033, 0.029, 0.040, and 0.026, respectively, greater than those of previous techniques, demonstrating that the proposed approach may enhance the quality of synthetic pictures. The PSNR value of the technique in this research is significantly enhanced when compared to the MAE and SSIM indicators. The PSNR values of the method in this work have been improved by 0.575 dB, 0.056 dB, 0.109 dB, and 0.257 dB, respectively, in addition to the GAN model based on residual U-Net. The method may be observed to increase the quality of the synthetic picture to some degree. The PSNR value of the method generated in this research is lower than the GAN model based on residual U-Net. This might be because PSNR is an error-sensitive picture quality rating statistic that ignores the human eye's visual features. As a result, the picture quality it reflects does not always match the image quality witnessed and verified by the human eye.  Figure 8 shows the quantitative evaluation of SSIM.

RETRACTED

As a consequence, the method in this study may improve the quality of the synthesized image and increase the edge synthesis impact of the picture by integrating the qualitative and quantitative findings of the experiment.

## 5. Conclusion

Aiming at the problems of blurred edges and low signal-to-noise ratio of synthetic results in cross-modal synthesis tasks of medical images, this paper proposes a cross-modal PET image synthesis method that fuses initial residual modules and generative adversarial networks. The authors provide a cross-sectional method that combines generative adversarial networks with residual modules. The method reduces the number of parameters and enhances the generator's capacity for feature learning by incorporating an improved residual initial module and attention mechanism. The discriminator uses a multiscale discriminator to improve discriminant performance. To better preserve visual contrast, a multilevel structural similarity loss is incorporated into the loss function. The algorithm is contrasted with the common algorithms using the ADNI data set. The experimental results show that the MAE index of the synthetic PET picture has decreased while the SSIM and PSNR indexes have increased. The experimental results imply that the suggested approach could preserve picture structural information while enhancing image quality in both subjective and visual metrics. By introducing improvements in the generator, the residual initial module and attention mechanism are used to improve the learning ability of the generator, and the multiscale discriminator is used to enhance the discriminative performance of the model. The comparative experimental results under the ADNI dataset show that the improved algorithm in this paper can preserve the image's structural information and contrast information. As a result, the generated image is visually closer to the actual print. However, there are still some shortcomings in this paper. For example, the medical images collected by instruments with different parameters have certain deviations. Furthermore, this paper uses the same preprocessing steps to process all data. Therefore, the data collection method and preprocessing method will have a particular impact on the experimental results. In addition, in the cross-modal PET composite image experiment, only the axial slice of the image is taken for the investigation, which cannot fully reveal the three-dimensional structural information of the brain. Therefore, different preprocessing methods and cross-modal synthesis methods for 3D PET images will be investigated next.

RETRACTED

### 5.1. Future Scope

Beyond the use of machine learning in medical imaging, we think the focus in the medical community may also be used to develop the overall computational attitude among healthcare practitioners and researchers, mainstreaming the discipline of computational medicine. The acceptance for further such systems will probably increase until there is enough high-impact application software based on mathematics, computer science, physics, and engineering entering the everyday workflow in the clinic. A new medical paradigm known as P4 medicine will most likely be made possible by the availability of biosensors and (edge) computing on wearable devices for monitoring illness or lifestyle, as well as an ecosystem of machine learning and other computing medicine-based technologies.

## Figures and Tables

**Figure 1:** Residual initial module structure [3]

**Figure 2:** Attention module [5].

**Figure 3:** Proposed framework.

**Figure 4:** Generator structure.

**Figure 5:** Comparative result.

**Figure 6:** Quantitative evaluation of MAE.

**Figure 7:** Quantitative evaluation of PSNR.

**Figure 8:** Quantitative evaluation of SSIM.

**Table 1:** Quantitative evaluation results of each algorithm.

Evaluation indicators	RIED-Net [5]	pix2pix [7]	Reset GAN [11]	pGAN [15]	Residual U-Net GAN [17]	Proposed algorithm
MAE	0.065 ± 0.030	0.063 ± 0.030	0.066 ± 0.030	0.072 ± 0.030	0.064 ± 0.030	0.062 ± 0.030
PSNR/dB	29.838 ± 0.815	30.357 ± 0.969	30.304 ± 0.642	30.156 ± 0.745	30.568 ± 1.056	30.413 ± 0.823
SIM	0.564 ± 0.133	0.637 ± 0.160	0.641 ± 0.736	0.630 ± 0.130	0.644 ± 0.150	0.670 ± 0.151

## Data Availability

The data shall be made available on request.
